# Estimation and Prediction of Hospitalization and Medical Care Costs Using Regression in Machine Learning

**DOI:** 10.1155/2022/7969220

**Published:** 2022-03-02

**Authors:** Ahmed I. Taloba, Rasha M. Abd El-Aziz, Huda M. Alshanbari, Abdal-Aziz H. El-Bagoury

**Affiliations:** ^1^Department of Computer Science, College of Science and Arts in Gurayat, Jouf University, Sakakah, Saudi Arabia; ^2^Information System Department, Faculty of Computers and Information, Assiut University, Assiut, Egypt; ^3^Computer Science Department, Faculty of Computers and Information, Assiut University, Assiut, Egypt; ^4^Department of Mathematical Sciences, College of Science, Princess Nourah bint Abdulrahman University, P.O. Box 84428, Riyadh 11671, Saudi Arabia; ^5^Basic Science Department, Higher Institute of Engineering and Technology, El-Mahala El-Kubra, Egypt

## Abstract

Medical costs are one of the most common recurring expenses in a person's life. Based on different research studies, BMI, ageing, smoking, and other factors are all related to greater personal medical care costs. The estimates of the expenditures of health care related to obesity are needed to help create cost-effective obesity prevention strategies. Obesity prevention at a young age is a top concern in global health, clinical practice, and public health. To avoid these restrictions, genetic variants are employed as instrumental variables in this research. Using statistics from public huge datasets, the impact of body mass index (BMI) on overall healthcare expenses is predicted. A multiview learning architecture can be used to leverage BMI information in records, including diagnostic texts, diagnostic IDs, and patient traits. A hierarchy perception structure was suggested to choose significant words, health checks, and diagnoses for training phase informative data representations, because various words, diagnoses, and previous health care have varying significance for expense calculation. In this system model, linear regression analysis, naive Bayes classifier, and random forest algorithms were compared using a business analytic method that applied statistical and machine-learning approaches. According to the results of our forecasting method, linear regression has the maximum accuracy of 97.89 percent in forecasting overall healthcare costs. In terms of financial statistics, our methodology provides a predictive method.

## 1. Introduction

The incidence of overweight and obesity has increased significantly in most countries in recent decades. Excess weight is associated with an increased incidence of many chronic diseases, including vascular disease, respiratory disease, osteoarthritis, some cancer, type 2 diabetes, and premature death. There is consistent evidence that an increased BMI is associated with higher health costs, and these costs are expected to increase as obesity. Modelling uses machine-learning methods, in which the machine learns from the data and uses it to forecast new data [1, 2]. The most commonly predictive analytic model used is regression [3–6]. The proposed model for accurate prediction of future outputs has applications in banking, economics, e-commerce, sports, business, entertainment, etc. A method used to forecast healthcare costs for BMI is based on several factors. Multiple linear regression is one of the statistical techniques for estimating the relationship among the dependent (target) and independent variables. The regression method is commonly used to develop a system based on a number of factors to predict the cost [5–11].

The regression analysis is performed to determine the relationship among two or more variables with cause-effect relationships and to make predictions for the topic using the relationships [12]. If regression used one independent variable, then it is known as univariate regression analysis, or else if it used more than two independent variables then it is known as multivariate regression analysis. Linear regression involves initially uploading the data and then analysing the data. Subsequently, the data are cut, and then, the data are trained and separated to create the model. At last, it will evaluate the accuracy. The main aim of regression is to develop an efficient technique for predicting dependent properties from a set of characteristic variables. A regression problem is the actual or continuous value of the output variables, that is, area, salary, and weight. Regression can be defined as a statistical method used in applications such as predicting the healthcare costs. Regression is used to predict the relationship among the dependent variable and set of independent variables. There are various types of regression techniques available namely simple linear regression, multiple linear regression, polynomial regression, support vector regression, and random forest regression [13].

Fast-growing healthcare costs have become a significant challenge in several developed countries. Existing evidence suggests that healthcare costs have accumulated among a large number of BMI. Even though experiments have attempted to develop accurate models for predicting healthcare costs for BMI, their effectiveness is excellent due to the lack of detailed clinical information in the data used to create complex intervals and prognostic models. Numerous studies on more costs for obesity patient prognostic models have relied on self-report data and electronic health data from claims [14]. Data from laboratory tests are defined—these, more granular and detailed clinical information, lead to improvements in the prognostic model. A recent survey by health research program and claim data shows that there is an improvement in the performance of the machine-learning-based predictive model for health costs for obesity. Still, many insurers and providers worldwide are actively seeking an approach that can accurately predict obesity BMI [15].

However, despite the potential value of advanced machine-learning approaches for risk prediction, payers and providers still rely heavily on linear regression to manage and adapt their patient population [16, 17]. The slow adoption of advanced machine-learning techniques may be partly explained by the lack of familiarity with risk stabilization analysts with such techniques and the combination of complex interpretation and results required in practice. Machine-learning regression models are within the framework of standard linear regression and perform some sophisticated but less explicit machine-learning techniques [18, 19]. This study focused on fine linear regression models, which conducted a complete comparison of penalty regression with linear regression in forecasting overall health costs, which was not reported in the previously published literature. The major focus of this study is to estimate the health costs incurred due to obesity in the population.

The rest of this study is formalized as follows: Section 2 defines the related works on estimating the healthcare costs using various methodology methods.  Section 3 designates in detail the workflow of the proposed algorithm.  Section 4 represents the experiments with results and comparison graphics with existing works and its discussion. Finally, Section 6 concludes the study.

## 2. Related Work

Some of the recent literature that describes the various mechanism of estimating the costs of physical healthcare is summarized below. In [20], unplanned 30-day readmissions are a common occurrence among congestive heart failure (CHF) patients, posing major health concerns and increasing healthcare costs. It is critical to implement tailored treatment programs for high hazard patients of readmission in an attempt to prevent readmissions and lower healthcare costs. This necessitates recognizing high individuals at the time of hospital release. They constructed and evaluated a deep learning network to predict 30-day unplanned readmission using actual information from over 7,500 CHF patients hospitalized in Sweden. Using specialist characteristics and situational integration of medical knowledge provides a cost-sensitive implementation of the long short-term memory (LSTM) neural net. Using both machine-derived and professional characteristics, including frequent patterns, and resolving the issue of class imbalances, this research focuses on important parts of an EHR-driven forecasting system in a single framework. We assess each element's impact on forecasting effectiveness (F1 measure, ROC-AUC) and price benefits. In at least 2 evaluating criteria, it shows that the technique with all critical features outperforms the simplified approaches in terms of discriminating capability. Researchers also propose a basic economic assessment to predict annual income if high-risk patients are provided tailored therapies.

Patients with heart failure (HF) require precise hazard classification to implement tailored therapies focused on enhancing their efficiency of living and results [21]. To assess the economic benefit of complementing claim-based forecasting analytics with electronic medical record (EMR)-derived data and to contrast machine-learning techniques to conventional logistic regression in forecasting critical results in patients with HF, healthcare patients with HF from 2 healthcare professional systems in Massachusetts, Boston, were included in predictive research with a one-year follow-up duration. “Providers” comprise therapists, various medical professionals, clinicians, and their organization including the network. Logistic regression, gradient boosted modelling, regression trees, random forests, least absolute shrinkage, classification, and selection operation regression were used to predict all-cause morbidity, top cost decile, HF hospitalization, gradient boosted modelling, and home days loss larger than 25%. Information from network 1 was used to educate all algorithms, which were then evaluated in network 2. The area under high accuracy curves (AUPRCs) and overall value estimations from decision curves were obtained after choosing the best effective modelling strategy depending on the Brier score, calibration, and discrimination.

The goal of this study was to evaluate the effectiveness of machine-learning methodologies for predicting healthcare expenses connected with spinal fusion in aspects of gains or losses in Taiwan Diagnosis-Related Groups (Tw-DRGs) and to use these techniques to investigate the major features connected with spinal fusion medical costs. Methods: a data collection was gathered from a healthcare facility centre in Taoyuan, Taiwan, containing data on Tw-DRG49702 patients (without problems or comorbidity; posterior and other spinal fusion). Weka 3.8.1 was used to forecast using random forest, support vector machines, Naive Bayesian, C4.5 decision tree, and logistic regression approaches [22, 23]. The research showed that the random forest approach may be used to estimate the healthcare expenditures of Tw-DRG49702 and that it can help institutions improve the financially operational effectiveness of this procedure.

Because of the ageing populations and enhanced therapy of fundamental conditions, cardiac arrest is among the most complicated chronic disorders with a higher incidence. The incidence is projected to gradually climb, reaching 3% of the population in Western countries [24]. It is the leading reason for hospitalizations in people aged 65 and above, leading to substantial expenses and a significant societal effect. In the therapy of HF, the present “one-size-fits-all” strategy does not produce the optimal results for all patients. These facts pose a serious danger to the proper treatment of heart failure patients. It will take an unconventional method from a unique perspective on health care. We offer a unique forecasting, preventive, and personalized healthcare strategy, in which patients are actually in charge of their care, aided by a user-friendly online form that employs artificial intelligence (AI). This technique study outlines the demands in HF care, as well as the necessary paradigm shift and the factors necessary to make it happen. A digital physician is being developed through an exciting combination of medical and high-tech partners from patient coaching, serious gaming, North-West Europe, artificial intelligence, and combining state-of-the-art HF health care. The findings are intended to improve and customize self-care, in which patients conduct routine care chores without the intervention of healthcare experts, allowing them to focus on more difficult problems. This innovative approach to health care will lower prices per patient while increasing results, ensuring the long-term viability of top-tier HF health care.

In [25], DRG codes are useful for price tracking and allocation of resources since healthcare operators obtain predetermined levels of compensation for certain treatments under diagnosis-related group (DRG) payments. Coding, on the other hand, is usually done after the fact, after the patient has been discharged. They want to use normal medical text to forecast DRGs and DRG-based case mix index (CMI) at initial inpatient admission to forecast hospital costs in an acute context. Without manual coding, a deep learning-based natural language processing (NLP) method is tested to forecast cost-reflecting weights and per-episode DRGs on 2 cohorts (paid by All Patient Refined (APR) DRG or Medicare Severity (MS) DRG). In fivefold cross-validation trials on the first day of ICU admission, it attained macro-averaged area under the receiver operating characteristic curve (AUC) scores of 0•871 (SD 0•011) on MS-DRG and 0•884 (0•003) on APR-DRG. When applied to hypothetical patient populations to predict average cost-reflecting weights, the algorithm improved over time, yielding absolute CMI errors of 12•79 (2•31%) and 2•40 (1•07%) on the first day, correspondingly. Because the system can adjust to changes in admission time and cohort size while requiring no additional manual coding, it has the potential to aid in cost estimation for active patients and enable improved functional outcome in hospitals.

## 3. The Proposed Method Based on Linear Regression

Linear regression is one of the most common supervisory machine learning statistical analysis techniques [26]. It is commonly used to find linear correlations between two or more responses and predictive variables. The technique is divided into two types depending on the number of variables in the model such as simple linear regression and multiple linear regression. A response variable corresponding to a predictive variable is simple linear regression. Whether more than two response variables correspond to predictive variables is known as multiple linear regression as shown in Figure 1. This work used linear regression to study the relationship among total maintenance and other properties in datasets to obtain the properties most affected by the total cost of maintenance. 75% of the data in the dataset were trained, and 25% of the data were tested. Then, Pearson's correlation coefficient (PCC) for each simple linear regression sample was calculated. The PCC is determined and calculated by the following equation to find the parallel variability and strength of a linear regression relationship between two factors:

(1) $$\begin{array}{c} Y_{i}^{\prime }=f_{n}\left(X_{i}^{\prime },\;\beta_{p\;}\right)+\;e. \end{array}$$

Here, *X*_*i*_′  and *y*_*i*_′  represent the independent variable and dependent variable; *f*_*n*_ represents the function; *β*_*p* _ represents the unknown parameters; and *e* represents the error terms. The most commonly used measurements to estimate the performance of a linear regression are the root mean square error (RMSE), the mean absolute error (MAE), and the mean square error (MSE) [26]. The following equations denote the error deviation for regression:

(2) $$\begin{array}{c} \text{RMSE}=\;\sqrt{\frac{\sum_{j=1}^{M}\left(y_{i}-\;y_{i}^{\prime }\right){\;}^{2}}{M}}, \end{array}$$

(3) $$\begin{array}{c} \text{MAE}=\;\sum_{i=1}^{N}\frac{x_{i}-x}{N}, \end{array}$$

(4) $$\begin{array}{c} \text{MSE}=\frac{1}{N}\sum_{j=1}^{N}\left(y_{i}-\;y_{i}^{\prime }\right){\;}^{2}. \end{array}$$

These regression measurements are constant variables and standard measurements for determining sample accuracy.

### 3.1. Regression's Role in Predicting the Costs

Clinics are encouraged to find more meaning in the substantial amount of data they generate and store each day [27]. Regression provides useful predictive accuracy and value for machine-learning clinics' databases with useful methods, features, and structures and contributes to a variety of strategies. The regression method aims to identify the possibility of improving results based on the predictive value of large-scale datasets for annual health costs. This is evidence of effectiveness in dealing with priority tasks, which defines that behaviours have the maximum tendency to cause preferred outcomes.

### 3.2. Steps for Applying Regression to Datasets

The database used here is a collection of medical expense personal data, which contain anonymous information about people. These data will act as a method learning object to generate functional information. In Table 1, the attributes such as BMI and age are continuous variables, and the attributes such as smoker and sex are categorical variables:

- The next step is data exploration and preparation, and the quality of any machine-learning program is largely based on the quality of the data it uses. This stage requires more human intervention in the machine-learning process. Frequently cited statistics show that 80% of efforts in machine learning are dedicated to data. Most of this time is spent learning more about data and its nuances throughout an exercise known as data analysis.
- Then, a model on the data is trained. The specific machine-learning task will announce the selection of the suitable method, and the method will denote the data in the form of a model.
- Subsequently, the model performance is evaluated. It is important to evaluate how well the method has learned from its past experience as each machine-learning model results in a biased solution to the learning problem. Depending on the type of model used, the accuracy of the sample can be estimated using the experimental database.
- Finally, the performance of the model is improved. It is necessary to use advanced techniques to increase the performance of the model if better performance is required. Each time, an entirely different type of model may have to be changed. After completing these steps, if the model appears to be operating acceptably, it can be used for its intended purpose. This model can be used to provide score data for forecasting, for financial data forecasting, to generate relevant insights for marketing or research, or to automate tasks.

### 3.3. Dataset Description

We intended to forecast a patient's healthcare costs for the coming year depending on their insurance payment statistics and previous healthcare data. Tsuyama Chuo Hospital contributed the healthcare record information. These documents come from healthcare insurance applications that the hospital is required to submit to the administration. Every patient is recognized by an individual identity (ID) in these reports, which include the patient's conditions, medications, operations, and payment details [28]. This claim's comprehensive paperwork can be obtained on the relevant website. We were able to retrieve the following information using this information:

- Patient demographics include age and gender.
- Patients' characteristics include their body fat percentage, height, weight, and waist circumference.
- Health care verifies the outcomes of a patient's healthcare check-up tests. Every testing is assigned a code, and the outcome should be provided. Blood pressure (BP) and creatinine levels are two instances. There are 25 various categories of tests, as well as the date that they were gathered.
- Prognosis: a patient's ailment is diagnosed using ICD-10 codes and is tracked by date.
- Payment details: for every session or hospital stay, every patient was assigned a score. This result effectively corresponds to the expense of a patient payment, which is the figure we needed to forecast for the following years.

It has been demonstrated that predicting patients' healthcare costs solely based on medical data is difficult. Preceding healthcare expenses are the strongest predictor of future expenditures: a longer history of healthcare expenditures is considered to increase forecasting. Depending on this fact, it is easier to anticipate future healthcare expenses when patients' information is available for multiple periods. When attempting to forecast expenditures for a single year, at least a two-year history is required [29].

Patients' monthly histories were included in our database. Furthermore, since many patients only had limited claims per year, there are several missing data. As a result, we decided to arrange claims by year to reduce the number of missing information. This technique did not work out as planned because many patients only had data [30]. We next screened out these patients, leaving only those with clinical history. The fundamental characteristics of these patients are shown in Table 2.

Figure 2 forecasts every patient's scores for the following year. These scores are directly proportional to the amount of cost a patient spent on health care. The range of patient values is depicted in the graph. As anticipated for healthcare expenses, the scores exhibit all similar patterns as indicated previously, with a spike at zero and a lengthy right-hand tail.

It has been claimed that using medical characteristics produces similar results as using solely expense predictions. Although the fact that medical record appears to have little effect on forecast accuracy, we choose to maintain it because it can enhance the range of variables in the algorithm, which might enhance vector differentiation. Every resource accessible as characteristics was used to encode a patient's history. Demographics, health check-up results, ICD-10 diagnostic groupings, real score, and preceding score are the inputs [31, 32]. The patient's vector is described in full in the table. We employed all of the parameters listed in the table as input vectors, with the exception of the real score, which was used as our target attribute.

### 3.4. Training Phase

We must determine the ideal hyperparameters of our system for a forecast to adapt as closely as feasible to its true value. The weights of every dimension used in the distance function and *g* in the discount function are these parameters. For the training process, we used the gradient-based methods since they have a strong mathematical foundation for achieving optimal results.

The gradient descent technique is an automated approach for minimizing or maximizing a target function by optimizing variable values. As our objective parameter, we used the mean absolute error (MAE), which is calculated as follows:

(5) $$\begin{array}{c} \text{MAE}=\;\frac{1}{n}\overset{n}{\underset{i=1}{\sum }}\left\|y_{i}\right.-\left.{\hat{y}}_{i}\right\|. \end{array}$$

The target is to minimize the values of the MAE equation, which is dependent on the variable *v*_*t*_ that could be either *γ* or *ω*. The following equation gives the updated value of *v*_*t*_, termed *v*_*t*+1_ as follows:

(6) $$\begin{array}{c} v_{t+1}=v_{t}-\propto \frac{\partial \text{MAE}}{\partial v}. \end{array}$$

This technique offers us a series of numbers for *v*_0_, ..., *v*_*k*_ that minimizes the MAE, with the first value for *v*(*i*.*e*.,  *v*_0_) generally chosen at random. During the training phase, we use all of the remaining *N* − 1 patients in *L* as evidence to try to forecast the expense of every patient *p*_*i*_ in the training set L. An epoch is an execution that computes forecasts for every '*N*′ patient; the gradient descent approach accumulates by completing repeated epochs.

### 3.5. Time Optimizing in Computing

A prediction's computing duration scales linearly with the size of the training phase. To find the mass of vectors of dimension *m* in a database with a training dataset of size *n*, we must firstly use the discounting function, which has a *O*(*m*) complexity. With the training set, we can estimate any discounting functions of the input vector in *O*(*mn*). Then, we can estimate *K* (9), which requires *O*(*mn*). for every output series and *O*(*mn*) for the accumulation; thus, we can estimate *K* in *O*(*mn*). time. Lastly, we require the discounting function, *K*, and a product series to get the mass, so we estimate the weights of the input vector (8) while keeping *O*(*mn*). Therefore, given *O*(*mn*). complexity, we could obtain the forecast.

According to reference, a *K*-nearest neighbour technique could be used to accelerate up calculation without sacrificing efficiency. For the actual closest neighbour's searches depending on product quantization, we used [33] methodology. Using this technique, we can generate indices for the *K*-nearest searches in time *O* (*mn*+*Kn*) within the training step. The weights of the *K*-nearest neighbours, which will be estimated in *O* (*Km*), are thus all that is required for a fresh forecast; the other weights are presumed to be null. Whenever the algorithm has been trained, the prediction's complexity is *O* (*Km*).

### 3.6. Interpretability

The IEVREG is a framework that is accessible. For every forecasting we generate, we could calculate the proportion (mass) of every element of information in the testing phase L. As a result, we have a complete understanding of how the anticipated quantity is calculated. This prototype is already interpretable, but to make it completely understandable, we will write a system of regulations for every forecast using the weights from the training dataset and the masses of every dimension gained all through the training step [34]. The idea is to calculate how much every piece of proof adds to the forecast. Firstly, using the weights of the existing N1 patients in the training dataset, we establish a system of regulations for each of the patients in the training phase for forecasting. Using the weights of the remaining N1 patients in the phases and the weights of the dimensions, we firstly build a system of regulations for each of the patients in the training phase [35, 36]. The limits of the measurements for each of the input characteristics, as well as their weights, are encoded by these principles. The algorithm then chooses the patients in the training phase who are the most identical and combines their principles to generate a new collection of criteria for that forecast.

We use a tiny healthcare coverage database only with 5 characteristics as input to demonstrate how we get the regulations with the IEVREG framework.  Table 3 shows the 5 data inputs (measurements) and the anticipated result for the healthcare expenses.

We used only the 60 closest neighbours to forecast this patient's result. The most significant principles (greater values) for expense forecasting are then obtained, as illustrated in Table 4. These are the limits and parameters that the patients have in common with the patients in the training phase.

We could see how a patient's expense projection is interpreted in Table 4. Low weight is associated with age in the IEVREG framework, while higher weight is associated with others. As a result, the method seeks out individuals with identical genders, BMIs, children, and smoking statuses, while ignoring age.

Algorithm 1 represents the steps of the linear regression model.

The flowchart for the proposed linear regression model is shown in Figure 3.

## 4. Results and Analysis

The average annual rates and costs of consultations, tests, and prescription items were estimated by BMI category at the time of recruitment as shown in Figure 4. Percentage differences in rates and average annual costs were calculated for women with a BMI greater than 2 kg/m^2^ and a BMI greater than 20 kg/m^2^, both overall and according to the type of drug use. All models were evaluated using semi-possible generalized linear models with variations such as record link and Poisson. At the beginning of each year, annual expenses are estimated in subgroups defined by alcohol consumption, socioeconomic status, smoking level, educational qualifications, and strenuous exercise in recruitment [37]. The diversity of the proportional increases in annual costs among the types of each subgroup was estimated using the chi-square test.

The mean absolute error, moreover, is ineffective for comparing outcomes with costs stated in various dollars, so we will use the mean absolute percentage error (MAPE), a customized absolute error in which the MAE is reduced by the mean cost and calculated as follows:

(7) $$\begin{array}{c} \text{MAPE}=\;\frac{\left(1/n\right)\sum_{i=1}^{n}|\left|y_{i}-{\hat{y}}_{i}\right||}{m}. \end{array}$$

Here, ${\hat{y}}_{i}$ is the estimated output for parameter *y*_*i*_ and *m* is the mean of variable *y*, denoted as follows:

(8) $$\begin{array}{c} m=\frac{1}{n}\sum_{i=1}^{n}y_{i}. \end{array}$$

We will also use additional metric, the *R*2, which reflects how closely we are to the true cost curve and is defined as the Pearson correlation among projected and real healthcare costs. The following formula is used to determine this significance:

(9) $$\begin{array}{c} R^{2}=1-\frac{\sum_{i=1}^{n}{\left(y_{i}-{\hat{y}}_{i}\right)}^{2}}{\sum_{i=1}^{n}{\left(y_{i}-m\right)}^{2}}. \end{array}$$

## 5. Discussion

We provided a novel linear regression technique that can simply demonstrate the purposes for producing a certain forecast regarding potential healthcare expenses, which is a useful capacity in the medical field. We evaluated its outcomes to the forecasting produced by the finest algorithms from the analysed research and reported to see how well it predicted. The linear regression is what we are talking about here. When we compare the outcomes of previous designs for the cost of healthcare forecasting approach, we can see that our system is more efficient, demonstrating that a more explicit approach for an issue such as healthcare cost forecasting is conceivable [38–40]. Our research, on the other hand, clearly reveals that healthcare spending is highly connected inside the Medicare program. There are approximately numerous people enrolled in the program. This finding could lead to preventive measures. Autocorrelation shows an inherent methodology that could be influenced by variables that can be changed. As a result, clinicians can use more accurate machine-learning algorithms to target these therapies to the proper HCHN group. There are a few flaws in this research. Initially, we performed the research within the context of a single state's Medicare system. The outcomes might differ depending on the state or kind of payer. Secondly, only general-purpose machine-learning algorithms were used. Certain customized versions might function optimally. Thirdly, the prediction algorithms offer no direction on the preventive characteristics that should be considered when developing treatments. Lastly, determining overall health solely based on claim statistics is restricted. Further input resources, such as descriptive elements of electronic health records (EHRs), illness intensity assessments, and socioeconomic determinants of health care, might well be required. A few of these restrictions will be addressed in the forthcoming research. We intend to broaden the scope of the study to include various sorts of healthcare initiatives. We will additionally collect the abovementioned extra data to assess predicted effectiveness [40]. We will also work with physicians and policymakers to make the algorithms more medically applicable using domain expertise to effectively target risk reduction actions.

## 6. Conclusion

We provided a new linear regression that can easily demonstrate the reasons for producing a certain forecast regarding potential healthcare expenses, which is a useful capacity in the healthcare area. The linear regression algorithm is used to estimate the healthcare costs of the patients such as obesity (BMI) using certain devices such as smartphones and smart devices. For estimation, by the use of linear regression, supervised learning performs more accurately. By providing comprehensive evidence, regression methodology can be effectively used for prognosis in conjunction with the dataset. The domain and time accuracy will determine the prediction model and the estimation of healthcare expenses. The proposed method reduces the risk of overfitting, and also, training time is less. This method is effective in estimating the healthcare costs of patients with an accuracy rate of 97.89%. The extensive tests on a real-time world database have confirmed the efficiency of our method.

## Figures and Tables

**Figure 1:** Block diagram for the proposed model.

**Figure 2:** Graphic representation of cost range for patients' score.

**Figure 3:** Flowchart for estimating the healthcare costs.

**Figure 4:** Healthcare expenses attributable to obesity and overweight between people on a yearly basis.

**Algorithm 1:** Linear regression (LR).

**Table 1:** Healthcare attributes and their specifications.

Attributes	Specifications
BMI	Body mass index
Age	Primary beneficiary age
Sex	Gender (male/female)
Smoker	The one who smokes affected by the obesity
Children	Number of children under BMI
Costs	Individual healthcare costs of the respective person

**Table 2:** Patients' characteristics and their predicted value.

Statistics	Predicted value
Total no. of patients	24,353
Mean value for expenses	10,538
Mean (age)	46.08
Male (%)	47.48
Female (%)	50.30

**Table 3:** Details of the patients.

Gender	BMI	Smoker	Age	Children	Actual value	Forecasted value
Female	29.98	No	37	1	6245	7154
Male	32.12	No	40	2	6725	7540

**Table 4:** Estimated values.

Gender	Estimated values	Weights
Male	30.6530 < BMI < 31.8560	0.45
	Gender = 0.0	0.45
	Children = 0.0	0.45
	Smoker = 0.0	0.45
	39.2016 < age < 40.2451	0.22
Female	28.5421 < BMI < 29.7451	0.39
	Gender = 0.0	0.39
	Children = 0.0	0.39
	Smoker = 0.0	0.39
	36.2016 < age < 37.2452	0.19

## Data Availability

The data used to support the findings of this study are available from the corresponding author upon request.
